This article has been retracted.

# MiR-27a promotes the autophagy and apoptosis of IL-1β treated-articular chondrocytes in osteoarthritis through PI3K/AKT/mTOR signaling

**DOI:** 10.18632/aging.102194

**Published:** 2019-08-27

**Authors:** Chen Cai, Shaoxiong Min, Bo Yan, Wen Liu, Xiao Yang, Liuxun Li, Ting Wang, Anmin Jin

**Affiliations:** 1 Department of Spine Surgery, Zhujiang Hospital, Southern Medical University, Guangzhou, Guangdong, China; 2 Department of Spine Surgery, The Third Affliated Hospital of Southern Medical University, Guangzhou, Guangdong, China; 3 Department of Cell Biology, School of Basic Medical Science, Southern Medical University, Guangzhou, Guangdong, China

**Keywords:** osteoarthritis, apoptosis, autophagy, miR-27a, PI3K

## Abstract

Osteoarthritis (OA) is a common degenerative joint disorder, which involves articular cartilage degeneration as well as joint inflammatory reactions. The recent studies have identified microRNA (miRNA) as one of the epigenetic mechanisms for the regulation of gene expression. Here we aim to reveal the role of miRNA in the regulation of gene expression in articular chondrocytes and its significance in the OA pathogenesis. In the present study, miRNA profiling was performed using OA cartilage and normal healthy cartilage tissues. As compared to their levels in normal cells and tissues, miR-27a expression was found to be upregulated in OA cartilage and IL-1β-treated articular chondrocytes. TUNEL staining, as well as flow cytometry with Annexin V-FITC/PI double labeling indicated that miR-27a inhibition reduced the apoptosis of IL-1β-treated articular chondrocytes. Bioinformatics prediction and the dual-luciferase reporter assay indicated that miR-27a targeted the 3′-UTR of the *PI3K* gene to silence it. The PI3K mRNA level in OA cartilage and IL-1β-treated articular chondrocytes was also downregulated, comparing with normal cells and tissues. Transfection of chondrocytes transfected with the miR-27a inhibitor upregulated the PI3K expression. This study demonstrated miR-27a is a regulator of the PI3K-Akt-mTOR axis in human chondrocytes and could participate in OA pathogenesis.

## INTRODUCTION

Osteoarthritis (OA), a frequently seen degenerative joint disorder, is associated with pain, as well as joint malfunction [1]. OA displays the consistent degeneration of articular cartilage, causing the imbalanced generation and degeneration of articular chondrocyte ECM (extracellular matrix) [2]. The essential feature of OA is that the generation of aggrecan, as well as type II collagen is repressed [3, 4], while the generation of matrix-degenerating enzymes such as matrix metalloproteinase-13 (MMP-13) is reinforced [5]. Although human and animal researches have widely reported abnormal gene expression in OA articular chondrocytes led to its pathogenesis [6], the regulatory mechanism for the expression of these genes in articular chondrocytes remains to be elucidated. Recently, microRNAs (miRNAs) that possess epigenetic-like properties in the regulation of gene expression have also been considered as one of the epigenetic mechanisms [7]. Furthermore, OA therapies appear far from satisfactory. Innovative targets of OA, such as genes participating in OA generation, have been revealed with the help of genetic networks, and epigenetic, as well as miRNA-based methods [1].

The role of epigenetic regulation of gene expression to the development of OA has recently been widely reported [8, 9]. Numbers of miRNAs have been identified to be involved in the pathogenesis of OA in recent epigenetic studies. miRNAs may directly bind to catabolic and anabolic mRNAs to regulate their expression at a post-transcriptional level in cytoplasm with a complimentary sequence to induce cleavage and degradation, or block translation [10, 11]. MiRNAs are a conserved group of small RNAs consisting of 20–22 nucleotides that modulate the post-transcriptional expression of mRNAs via binding to their 3'-UTRs, thereby causing mRNA degeneration and the suppression of their translation [12]. For example, the functions of some crucial signaling pathways, including the NF-kappaB pathway [13, 14], Wnt/beta-Catenin pathway [15], SIRT1/p53 pathway [16], and SDF1/CXCR4 pathway [17], were demonstrated to be regulated via chondrocyte miRNAs involved in the development of OA. MiR-27a has been recognized as one of the most prolific miRNAs identified, considering its contribution to the modulation of multiple biological reactions [18], as well as the pathogenesis of various diseases, such as pancreatic cancer [19], gastric cancer [20], human hepatocellular cancer [21], and OA [22], mainly caused by its capability to target multiple oncogenes. Moreover, in the pathogenesis of various types of diseases, reduction of miR-27a expression has been found to be related to a worse prognosis [23].

Previous study has demonstrated that MiR-27a regulates apoptosis in nucleus pulposus cells by targeting PI3K [24]. In our study, the data revealed that the miR-27a level was remarkably elevated in OA cartilage, as well as IL-1β-treated articular chondrocytes, compared to normal cartilage or untreated chondrocytes. Moreover, miR-27a was predicted to target the 3′-UTR of the *PI3K* gene, proving the direct interaction between PI3K mRNA and miR-27a. Functional evaluation confirmed that miR-27a reduced the IL-1β-triggered apoptosis and autophagy of articular chondrocytes. Inhibition of miR-27a increased the expression of PI3K, and activated its downstream components Akt and mTOR. Given these findings, miR-27a may potentially be used to diagnosis and treatment of OA.

## RESULTS

### MiR-27a is upregulated in OA cartilage, as well as IL-1β-supplemented articular chondrocytes

To elucidate the contribution of miRNA to OA development, miRNA microarray analysis of OA samples and normal healthy samples was performed. We found that the miR-27a expression was remarkably increased in OA cartilage samples, compared to healthy controls (Figure 1A, 1B). Increasing evidences support a vital role for miR-27a in modulating polymorphisms, tumorigenesis, proliferation, apoptosis, invasion, migration and angiogenesis [22], therefore, miR-27a was chosen for further validation and elucidation. To confirm these data, Q-PCR analysis was performed for determining the expression of miR-27a in the OA specimens (n=20) and control samples (n=10). The miR-27a expression was found to be increased in OA cartilage as compared to the expression level in the healthy controls (n=10) (Figure 2A). Additionally, we examined the miR-27a expression in IL-1β-treated chondrocytes. The SW1353 cells were treated with 5 ng/ml IL-1β at 0, 3, 6, 12, or 24 h prior to the evaluation of the miR-27a expression. IL-1β was able to notably promote the miR-27a expression in a time-dependent manner, in comparison to the untreated controls (Figure 2B), indicating that miR-27a could participate in OA-related processes.

**Figure 1:** **Microarray data.** (**A**) Volcano plot displaying the alteration of microRNA (miRNA; 2-fold increase or decrease) expression versus p, as detected by the microarray analysis of OA patients relative to healthy controls. (**B**) Different expression levels of a set of microRNAs in OA patients and healthy controls. Green, low expression levels; red, high expression levels.

**Figure 2:** **The miR-27a expression in OA cartilage and IL-1β-triggered chondrocytes.** (**A**) miR-27a expression in normal (n=10) as well as OA cartilage samples (n=20) were evaluated using Q-PCR. (**B**) Chondrocytes were treated with 5 ng/ml IL-1β for 0, 3, 6, 12, or 24 hours. The miR-27a expression was assessed via Q-PCR, and normalization to the levels of GAPDH. The results are described as the mean ± SD. *P < 0.05, **P < 0.01 vs. indicated group.

### MiR-27a inhibition increased the viability and repressed the death of IL-1β-treated chondrocytes via apoptosis and autophagy

To analyze the contribution of miR-27a to the proliferation and viability of IL-1β-treated chondrocytes, the cells were transfected with an miR-27a repressor. The Q-PCR data showed that the transfection with the miR-27a repressor led to an obvious decrease in the miR-27a levels (Figure 3A). The MTT assay revealed that the growth rate of chondrocytes was noticeably inhibited at 24, 48, and 72 hours following their stimulation with IL-1β, but the transfection of cells with an miR-126 inhibitor completely recovered the growth rate (Figure 3B). Furthermore, the aberrant downregulation of miR-27a expression also resulted in a noticeable increase in the colony numbers of IL-1β-treated chondrocytes, according to evaluations made via the soft agar colony formation assay; however, treatment with IL-1β impaired the cell proliferation (Figure 3C). These results suggested that miR-27a may have an inhibitory effect on the growth of IL-1β-treated chondrocytes.

**Figure 3:** **Contribution of miR-27a expression to the growth of IL-1β-triggered chondrocytes.** (**A**) Expression levels of miR-27a in IL-1β-treated chondrocytes that underwent transfection with the miR-27a inhibitor and miR-Scr were evaluated by Q-PCR. (**B**) The proliferation rate of IL-1β-treated chondrocytes was measured at 24, 48, and 72 h following their transfection using the MTT test. (**C**) Soft agar colony generation assay of IL-1β-treated chondrocytes transfected with the miR-27a inhibitor and miR-Scr. The lower panel indicates the number of colonies in each group. The results are described as the mean ± SD. *P < 0.05, **P < 0.01 vs. indicated group.

Considering that miR-27a inhibition restored the IL-1β-induced inhibition of the proliferation of chondrocytes, we hypothesized that miR-27a silencing may inhibit the apoptosis or autophagy of chondrocytes. Firstly, to test the effect of miR-27a on cell apoptosis, both TUNEL staining (Figure 4A) and flow cytometry with Annexin V-FITC/PI double labeling (Figure 4B) were performed, indicating notable apoptosis in chondrocytes treated with IL-1β, while the number of apoptotic cells decreased noticeably after transfection with the miR-27a inhibitor, compared to the untreated cells and cells that were transfected with miR-Scr. In addition, increased Bcl-2 levels and decreased Bax levels also indicated that miR-27a inhibition inhibited the IL-1β-induced cell apoptosis (Figure 4C)

**Figure 4:** **Downregulation of miR-27a expression repressed the apoptosis levels in IL-1β-triggered chondrocytes.** (**A**) TUNEL staining was performed to detect the number of dead cells in case of IL-1β-treated chondrocytes that underwent transfection with the miR-27a inhibitor and miR-Scr. Magnification, ×100. The apoptotic rate based on positive TUNEL staining in each group is displayed in the lower right panel. (**B**) FC was performed to assess the number of dead cells that were transfected with the miR-27a inhibitor and miR-Scr. The upper right quadrant of every plot represents the early apoptotic cells. The apoptotic rate analysis of IL-1β-treated chondrocytes in each group is presented in the lower right panel. (**C**) WB was performed to detect the expression of the apoptotic markers, Bcl-2 and Bax, in IL-1β-treated chondrocytes. The results are described as the mean ± SD. *P < 0.05 vs. indicated group.

Enhancement of autophagy in chondrocytes can delay the progression of osteoarthritis by affecting intracellular metabolic activity via regulating cell aging and death [25], therefore, we hypothesized that miR-27a inhibition mediated the autophagy of IL-1β-treated chondrocytes was also investigated. Hence that, IFA was performed to trace the location of the LC3B protein following miR-27a inhibition. At first, LC3B (green) was accumulated due to IL-1β treatment, while miR-126 silencing markedly reduced the number of LC3B dots (Figure 5A). MiR-27a inhibition reduced the autophagy rate of IL-1β-treated chondrocytes, as indicated by the decrease in LC3B biosynthesis and processing (reduced LC3B I and II levels), together with attenuated p62 degradation (two major indicators of the autophagic process) (Figure 5B). Transcription of p62 was evaluated using Q-PCR, and the results showed that its expression was inversely linked with the cellular miR-27a expression (Figure 5C). Collectively, these findings proved that miR-27a may increase the apoptosis and autophagy of IL-1β-treated chondrocytes, which is partially responsible for its inhibitory effect on IL-1β-treated chondrocyte proliferation.

**Figure 5:** **Downregulation of miR-27a expression repressed the autophagy in IL-1β-triggered chondrocytes.** (**A**) Twenty-four well plates were used to culture IL-1β-supplemented chondrocytes. The cells were first co-transfected for 36 h with the GFP-LC3B construct, as well as the miR-27a inhibitor/miR-Scr. The cellular location of GFP-LC3B was then evaluated via IFA (magnification, ×400). (**B**) WB was used to analyze the expression levels of LC3B and p62 in IL-1β-supplemented chondrocytes transfected with the miR-27a inhibitor. (**C**) Q-PCR was used to analyze the mRNA expression of p62 in IL-1β-treated chondrocytes transfected with the miR-27a inhibitor. The results were described as the mean ± SD. *P < 0.05, **P < 0.01 vs. indicated group.

### MiR-27a targeted the 3'-UTR of PI3K

Reportedly, the PI3K-Akt-mTOR axis was found to be related to the apoptosis and autophagy of different cell lines [26, 27]. Therefore, we determined the expression of PI3K in IL-1β-treated chondrocytes. PI3K protein and mRNA levels were both repressed in OA cartilage samples compared to the normal cartilage samples (Figure 6A, 6B). Furthermore, the bioinformatics analysis suggested that miR-27a may target the 3'-UTR of PI3K (Figure 6C). A direct interaction between miR-27a and the 3'-UTR of PI3K was detected by performing the DLRA. The above findings revealed that luciferase function was inhibited following the transfection of the cells with the miR-27a mimic, which showed a 90% interaction with the 3'-UTR of PI3K, compared to the case for the control groups (Figure 6D).

**Figure 6:** **MiR-27a directly targets PI3K.** (**A**) PI3K expression in normal (n=10) as well as OA cartilage samples (n=20) were evaluated via Q-PCR. (**B**, **C**) Chondrocytes were treated with IL-1β (5 ng/ml) for 0, 6, 12, or 24 hours. The PI3K expression was assessed by Q-PCR and WB analyses. (**D**) Graphical representation of the conserved miR-27a-binding motif at the 3′-UTR of PI3K. (**E**) The DLRA was performed following the transfection of the cells with the luciferase reporter constructs that included either mutated (MU) or wild-type (WT) sequences of human PI3K 3'-UTR after transfection with the miR-27a mimic/miR-Scr. The luciferase activity was normalized to the β-galactosidase activity. Q-PCR (**F**) as well as WB (**G**) analyses were performed to assess the PI3K transcription and translation levels, as well as the Akt, phosphor-Akt, and mTOR protein levels, following the transfection of IL-1β-treated chondrocytes transfected with the miR-27a inhibitor and miR-Scr. The results are described as the mean ± SD. *P < 0.05, **P < 0.05 vs. indicated group.

We also analyzed the effect of the aberrant, downregulated expression of miR-27a on the PI3K expression in IL-1β-treated chondrocytes using Q-PCR and WB analyses. Protein and mRNA expression levels of PI3K were upregulated following transfection with the miR-27a repressor (Figure 6F, 6G). Additionally, PI3K upregulation activated the expression of its downstream components Akt and mTOR. These results demonstrated that the expression of PI3K and its associated pathways increased following the inhibition of miR-27a expression; miR-27a potentially targeted the 3'-UTR of PI3K.

### PI3K knockdown attenuated the miR-27a inhibition-mediated increase of the viability of IL-1β-treated chondrocytes

To determine whether PI3K silencing may reverse the impact of miR-27a on the viability of IL-1β-treated chondrocytes, PI3K transcription was silenced in chondrocytes that were co-transfected with the miR-27a inhibitor. Q-PCR and WB analyses were performed to confirm the change in the PI3K levels in cells (Figure 7A, 7B). We further showed that with the depletion of PI3K expression, Akt activation and mTOR expression were suppressed. Moreover, PI3K silencing inhibited the proliferation of IL-1β-treated chondrocytes, which was promoted by the miR-27a inhibitor, as estimated via the MTT assay (Figure 7C).

**Figure 7:** **Silencing the PI3K expression restored the impact of miR-27a inhibition on the growth of IL-1β-treated chondrocytes.** IL-1β-treated chondrocytes were co-transfected with the miR-27a inhibitor/miR-Scr and shRNA-PI3K/shRNA-NC. (**A**) The PI3K expression in cells after their transfection was assessed at the mRNA level by Q-PCR. (**B**) WB was performed to detect the Akt, phosphor-Akt, and mTOR protein levels in IL-1β-treated chondrocytes. (**C**) The proliferation rate of IL-1β-treated chondrocytes was examined at 24, 48, and 72 h following the transfection, utilizing the MTT test. **P < 0.01 vs. indicated group.

To evaluate the role of PI3K in the death of IL-1β-treated chondrocytes, apoptosis of IL-1β-treated chondrocytes was assessed via flow cytometry with Annexin V-FITC/PI double labeling. Aberrant downregulation of PI3K expression remarkably increased the number of dead cells, following transfection with the miR-27a inhibitor (Figure 8A).

**Figure 8:** **Silencing the PI3K expression increased the apoptosis and autophagy of IL-1β-treated chondrocytes, which were impaired by miR-27a inhibition.** IL-1β-treated chondrocytes were co-transfected with the miR-27a inhibitor/miR-Scr and shRNA-PI3K/shRNA-NC. (**A**) PI3K silencing restored the apoptotic levels attenuated by the miR-27a inhibitor. FC analysis and Annexin V-FITC/PI staining were performed to examine the number of early apoptotic IL-1β-treated chondrocytes at 36 h after their transfection. (**B**) WB was performed to analyze the expression levels of LC3B and p62 in IL-1β-treated chondrocytes. (**C**) Q-PCR was performed to analyze the mRNA expression of p62 in IL-1β-treated chondrocytes subjected to miR-27a inhibition and/or PI3K silencing. The results are described as the mean ± SD. *P < 0.05, **P < 0.01 vs. indicated group.

On the other hand, our data showed that PI3K silencing caused a significant upregulation of autophagy, as evidenced by increased LC3B processing and biosynthesis, as well as p62 degradation (Figure 8B). Q-PCR was then performed to examine the p62 transcription. Results showed that its expression was positively related to PI3K expression (Figure 8C). This indicates that PI3K silencing impaired chondrocyte proliferation via miR-27a-mediated apoptosis and autophagy.

### Effect of balA on autophagic flux induced by PI3K silencing

To further evaluate autophagic flux suppressed by miR-27a inhibition and induced by PI3K silencing, we determined whether miR-27a inhibition and PI3K silencing mediated regulation of LC3BII and p62 was affected by co-treatment with bafilomycin A (balA). WB analysis revealed that PI3K silencing effectively downregulated p62 expression in IL-1β treated chondrocytes, while co-treatment with bafA protected autophagic p62 from degradation (Figure 9A). However, no change was found in LC3B-II upon bafA co-treatment. This result indicates that PI3K mediated cell autophagic is completely reversed by autophagic inhibitor balA in L-1β treated chondrocytes.

**Figure 9:** **Effect of balA on autophagic flux induced by PI3K silencing.** (**A**) Autophagic flux was determined in IL-1β treated chondrocytes. Cells with inhibited expression of miR-27a and PI3K were co-treated with bafA for 12 hrs. Cell lysates were subjected to WB analysis using anti-p62, anti-LC3B and anti-GAPDH antibodies. (**B**) Annexin V-FITC&PI staining of IL-1β treated chondrocytes co-treated with BafA (100 nM) for 24 hrs. Data are representative of three independent experiments.

Furthermore, we next tested whether PI3K silencing induced apoptosis is dependent on autophagy. Chondrocytes were co-transfected with miR-27a inhibitor and shPI3K in the presence and absence of bafA, followed by annexin V-FITC&PI staining and flow cytometric detection of apoptotic cells. PI3K silencing in IL-1β treated chondrocytes resulted in varying but significant increase in annexin V positive cells. Co-treatment with bafA completely abolished PI3K silencing-mediated annexin V positivity in these cells (Figure 9B). Taken together, this data suggests that PI3K silencing induces apoptosis in an autophagic-dependent manner.

## DISCUSSION

Aberrant regulation of miRNA levels is closely involved in multiple diseases, including OA [28, 29]. A previous study has shown that miR-103, miR-377, miR-22, and miR-483 were upregulated, while miR-25, miR-26a, miR-337, and miR-299 were downregulated in OA cartilage, compared to the case in normal cartilage [30]. In addition, multiple miRNAs have been reported to modulate OA development. For instance, microRNA-142-3p represses chondrocyte death as well as inflammatory reactions of OA via the repression of the HMGB1-modulated NF-κB pathway [31], which is also repressed by miR-210 via targeting DR6, in OA [16]. Consequently, it is crucial to reveal genetic networks modulated via these miRNAs in OA. Our research proved that miR-27a expression was remarkably increased in OA cartilage and IL-1β-treated chondrocytes, compared to the case for the normal controls. It was thus, indicated that miR-27a is a promising contributor to OA generation.

A previous investigation has found that IL-1β plays a critical role in cartilage degeneration, which is associated with the etiology of OA [32]. Articular cartilage ECM mediates various biological reactions such as chondrocyte growth, differentiation, attachment, and viability, which are important for the recovery as well as the homeostasis of cartilage [33]. The continuous damage of cartilage ECM represses joint activity and contributes to OA development [3]. IL-1β was able to regulate the generation of ECM components of chondrocytes, including collagen type II and aggrecan [34]. Moreover, IL-1β mediates the production of MMPs in chondrocytes, such as MMP-1, MMP-3, and MMP-13, which destroys cartilage components [35]. According to these previous studies, we treated SW1353 cells with IL-1β in this study. We performed a series of analyses with miR-27a regulation to determine whether IL-1β regulated the major properties of chondrocytes. Our research discovered that IL-1β stimulation attenuated cell growth, and induced cell death and autophagy. In contrast, downregulation of miR-27a efficiently invalidated the IL-1β-induced inhibition of cell proliferation and activation of apoptosis and autophagy in chondrocytes. Thus, our research suggested that the downregulation of miR-27a might inhibit OA progression by ablating the influence of IL-1β.

Accumulating miRs may affect biological reactions via the modulation of their target agents. Previous research has demonstrated that miR-27a may target different genes, such as *DKK2*, *SFRP1* [36], *TLR4* [37], *FOXO1* [38], and *CASR* [39], which are all involved in the progression of different diseases. Using bioinformatics analysis, we predicted that miR-27a may target the conserved site of PI3K. DLRA results showed that PI3K directly interacted with miR-27a in 293T cells. PI3K and its downstream components (Akt and mTOR) are correlated with multiple biological processes [40–42], with phosphorylated Akt modulating various genes, especially pro-apoptotic factors, including Bcl-xL, Bcl-2, Bax, VEGF, and MMPs [43–45]. Previous research has also indicated that the PI3K-Akt-mTOR pathway may be associated with various aspects of autophagy [46–48]. A complicated group of pathways modulates autophagy. In this study, PI3K expression was found to be increased following miR-27a inhibition in IL-1β-treated chondrocytes, along with the reduction of apoptosis and autophagy; in contrast, PI3K silencing lead to the recovery of the apoptosis and autophagy that was triggered by the IL-1β treatment. Taken together, the results suggest that miR-27a may considerably contribute to OA development by modulating the PI3K-Akt-mTOR pathway.

In conclusion, the findings of our study suggest that the upregulation of miR-27a expression directly downregulated PI3K, causing apoptosis and autophagy in IL-1β-treated chondrocytes. Additional research on miR-27a could offer innovative insights into the mechanisms of, and therapies for, OA.

## MATERIALS AND METHODS

### Specimens

Cartilage specimens (human) were acquired from 20 OA patients who underwent total knee replacement surgery; cartilage from 10 traumatic amputees with neither OA nor rheumatoid arthritis were used as controls. Diagnosis of OA was made using the American College of Rheumatology criteria. All specimens were obtained from the Department of Spine Surgery, Zhujiang Hospital. Informed consent was acquired from every participant and the procedures were approved by the Ethics Committee of the Zhujiang Hospital, Southern Medical University.

### Cell cultivation

Human chondrosarcoma (SW1353) cells resemble chondrocytes phenotypically [49]; thus, they were utilized as a replacement for cartilage cells in order to examine the modulatory effects of miRNAs. SW1353 cells were purchased from the ATCC and were cultivated using DMEM containing 10% fetal bovine serum (FBS) and 1% penicillin and streptomycin under conditions of 5% CO_2_ at 37°C.

Cartilage samples were isolated and cut into small slices (0.5×0.5×0.5 cm^3^), and were subjected to 30 min of digestion with trypsin (0.1%, w/v) (Sigma) and 16 h of digestion with collagenase II (0.15%, w/v) (Sigma) at 37°C. The suspensions were filtered through a 100-μm nylon cell strainer (BD Falcon) and rinsed with DMEM (Hyclone) containing 10% FBS (GIBCO). T-75 culture flasks were utilized in order to culture the separated chondrocytes in DMEM containing 10% FBS (v/v), 100 μg/ml streptomycin (GIBCO), and 100 U/ml penicillin. Chondrocytes from the first passage were used for additional assays.

### Transfection

SW1353 cells underwent transfection with 100 nM of miR-Scr (5’-UGG AAU GUA AAG AAG UAU GUA U-3’) or miR-27a inhibitor (5’-AGG GCU UAG CUG CUU GUG AGC A-3’, RiboBio, Guangzhou, China) utilizing Lipofectamine 3000 reagent (Invitrogen), as instructed. Cells were activated using IL-1β or PBS for 24 h following transfection. The supernatants were harvested. Total RNA, as well as proteins acquired from chondrocytes were quantified to examine the expression of PI3K, phosphor-Akt, p62, miR-27a, Akt, mTOR, and GAPDH.

### miRNA array

Total RNA was isolated using the phenol-chloroform approach (Invitrogen; TRIzol; Thermo Fisher Scientific, Inc., Waltham, America). The RNA quality was evaluated by capillary electrophoresis (instrument provided by Agilent Technologies Inc., Santa Clara, America). Following small RNA sequencing, libraries were generated using the NEBNext Multiplex Small RNA Library Prep Set for Illumina (provided by New England BioLabs, Inc., Ipswich, America) as instructed. The libraries were quantified on the Agilent Bioanalyzer 2100 system using high-sensitivity DNA chips. Raw sequence files were subjected to quality control assessment using the FastQC quality control instrument. Adaptors were eliminated via Cutadapt (version 1.2.1) and sequences with lower quality were trimmed in order to prevent low-quality data. Clean miRNA reads were examined at the length of 21–22 nt and were compared to the reference sequences using the Bowtie software (provided by CGE Risk Management Solutions B.V., The Netherlands; version 2). Activities of various miRNAs were assessed using the miRDeep2 software (version 2.0.0.8). Differential expression sequencing was utilized in order to examine the differential expression and alterations between the specimens and control samples.

### Soft agar colony formation assay

The cells were transfected with the miR-Scr or miR-27a inhibitor. Two days after their transfection, the cells were resuspended in DMEM containing 10% FBS as well as 8mm top agar (0.4%) before being transported to 12-well plates including 0.5 ml bottom agar (0.5%). After 14 days, we selected three random regions in every plate to count the number of colonies.

### MTT assay

The MTT test was performed to assess the cell survival. First, 20 μl of MTT (0.5 mg/ml) was added to each well. Then, 100 μl of DMSO was added to each well; the samples were mixed for 10 mins to aid the dissolution of the formazan dye formed following the addition of MTT. The absorbance of each sample was then assessed at 490 nm using an Infinite M200 microplate reader (Tecan, Männedorf, Switzerland).

### Cell death assessment

Cell death was assessed using an annexin V-FITC and PI apoptosis detection kit. Following their transfection, the cells were resuspended in 20 μl of binding buffer; then, 5 μl of PI and 10 μl of annexin V-FITC was added to the cells. The samples were then incubated for 20 min in the dark. Flow cytometry (FC) analysis was performed to assess the cell death.

### TUNEL staining

To evaluate the alterations associated with cell death, TUNEL staining was performed using a TUNEL fluorescence kit (Roche, Basel, Switzerland) to stain the cells, apart from staining the nuclei with DAPI (1:5000, Beyotime, China). Cell death was determined by calculating the number of cells that showed positive TUNEL staining using a Laser Scanning Confocal Microscope (SP8, Leica, Japan).

### Immunofluorescence assay (IFA)

For the LC3B puncta assay, cells were transfected with GFP-LC3B expression constructs (Addgene). Images were recorded using a fluorescent microscope, as mentioned in a previous report [50]. The GFP puncta in 10 different microscopic fields were estimated.

### Western blotting (WB)

The cell lysis was performed using a protease suppressor cocktail (Roche) in a RIPA buffer (pH 8.0) containing NP-40 (1%), SDS (0.1%), Tris-HCl (50 mM), and NaCl (150 mM). A BCA Protein Quantitation Kit was employed for the quantification of proteins. These protein samples were isolated on SDS-PAGE gels (10%), and then, the protein bands were transferred onto PVDF membranes (0.45 μm). The membranes were then blocked for 60 min using PBST containing 5% BSA at an ambient temperature. Afterwards, these membranes were incubated for 60 min with specific primary antibodies at 4°C. The primary antibodies used were listed here: Bcl-2 ab (1:1000, ab59348, Abcam), Bax ab (1:1000, ab227754, Abcam), LC3B-I ab (1:500, ab48394, Abcam), p62 ab (1:2000, ab56416, Abcam), PI3K ab (1:2500, ab227204, Abcam), mTOR ab (1:1000, ab2732, Abcam), Akt ab (1:2000, ab8805, Abcam), pAkt ab(1:500, ab38449, Abcam), and GAPDH (1:5000, ab8245, Abcam) Then, the membranes were incubated with the secondary antibodies conjugated with Amersham ECL peroxidase: goat anti-rabbit IgG (1:5,000) or goat anti-mouse IgG (1:5,000) at an ambient temperature for another 60 min. The immunoreactivity was measured using a Super Signal West Femto Maximum Sensitivity Substrate Kit (provided by Thermo) on a C-DiGit Blot Scanner.

### RNA isolation and Q-PCR

Trizol reagent was utilized to separate the total RNA. The Roche Light-Cycler 480 Real Time PCR system was utilized in order to evaluate the transcription levels. GAPDH served as the internal reference. SYBR Green PCR Master Mix was used for qPCR (total reaction volume, 20 μL). The PCR was performed using the following temperature cycles: initial denaturation (10 min; 95°C), forty cycles of denaturation (15 s; 95°C), and extension (30 s; 72°C). Quantification was carried out using the 2^-ΔΔCT^ approach, and the expression levels of the tested genes were normalized relative to those of GAPDH (mean of the controls), while the levels of miR-27a were normalized to U6 controls. The sequences of primers used were listed as follows: miR-27a F: 5’-TCC GTG AGA GCT GGA AAA CC-3’, miR-27a R: 5’-TGG TTC TAA CTA ACT CCA GCC G-3’; p62 F: 5’-GCC AGA GGA ACA GAT GGA GT-3’, p62 R: 5’-TCC GAT TCT GGC ATC TGT AG-3’; PI3K F: 5’-AAC ACA GAA GAC CAA TAC TC-3’, PI3K R: 5’-TTC GCC ATC TAC CAC TAC-3’; GAPDH F: 5’-CAC CCG CGA GTA CAA CCT T-3’, GAPDH R: 5’-CCC ATA CCC ACC ATC ACA CC-3’.

### DLRA (dual-luciferase reporter assay)

Using the GV126 luciferase gene, the PI3K 3′-UTR sequence was amplified before its fusion with the constructs. The binding sites on the *PI3K* gene, apart from that for miR-27a, were ablated through site-directed mutagenesis; these samples served as the control. Thymidine kinase promoter (TaKaRa, Japan; pRL-TK vectors) and plasmids containing *Renilla* luciferase were used to normalize for transfection efficiency. 293T cells were co-transfected with the miR-27a mimics, as well as the negative controls utilizing the luciferase reporter vectors. The luciferase assay was then performed.

### Statistical analysis

The results were displayed as the means ± SDs. Differences between the groups were evaluated using 2-tailed Student’s t-test or ANOVA. P < 0.05 was considered statistically significant.
